# Lag-Based Filtered-Delay Multiply and Sum Beamformer Combined with Two Phase-Related Factors for Medical Ultrasound Imaging

**DOI:** 10.1155/2020/1503791

**Published:** 2020-08-28

**Authors:** Ke Song, Paul Liu, Dong C. Liu

**Affiliations:** ^1^School of Mathematics and Information Engineering, Chongqing University of Education, Chongqing 400065, China; ^2^Stork Healthcare Ltd., Chengdu 610041, China; ^3^Saset (Chengdu) Inc., Chengdu 610041, China

## Abstract

A novel adaptive beamformer named filtered-delay multiply and sum (F-DMAS) has recently been proposed. Compared to the delay and sum (DAS) beamforming algorithm, F-DMAS can efficiently improve the resolution and contrast. However, the DAS can still be seen in the expansion of DMAS. Therefore, we rearrange the pair-wised signals in terms of lag in DMAS and then synthesize a lot of new signals. Thanks to the relationship between the spatial coherence and lag, these new signals can be thought of as sorted by the spatial coherence. Thus, we apply two phase-related factors, the polarity-based factor (PF) and the sign coherence factor (SCF), which are evaluated based on new signals, to weight the output of DMAS. The two approaches are consequently referred to as LAG-DMAS-PF and LAG-DMAS-SCF, respectively. The results show that, compared to F-DMAS and DAS, our proposed methods can improve the resolution and contrast to some extent without increasing too much computational complexity. In the comparison between LAG-DMAS-PF and LAG-DMAS-SCF, the latter has better performance, but the former can better protect image details.

## 1. Introduction

Ultrasound imaging technology has been widely used for decades. The beamformer, as an important component in ultrasound imaging system, has made great progress and evolved from analog technology to digital technology [1, 2]. The delay and sum (DAS) beamformer, which is robust and simple to implement, is a popular technology. However, its performance, in terms of resolution and contrast, is not good [3]. Therefore, many researchers have proposed a lot of new methods, such as the minimum variance (MV) [3–5], the short-lag spatial coherence (SLSC) [6–9], the pixel-based beamforming [10, 11], and neural networks for beamforming [12, 13].

In addition to the methods we mentioned previously, a novel filtered-delay multiply and sum (F-DMAS) beamformer has been proposed for ultrasound B-mode medical imaging [14]. This method can enlarge the difference between coherent signals and incoherent signals through the multiplication of pair-wised signals. It shows that the resolution and contrast can be significantly improved in comparison with DAS [14]. Since then, a lot of researches on this algorithm have emerged. Park et al. [15] applied it to photoacoustic microscopy and introduced a method to simplify the computation. Matrone et al. [16] combined the F-DMAS with multiline transmission (MLT) to suppress the crosstalk artifact. Prieur et al. [17] analyzed the F-DMAS beamforming algorithm from statistics point of view and showed that the F-DMAS was more susceptible to signal coherence in comparison with the DAS. Matrone et al. [18] discussed the application of the F-DMAS beamforming algorithm to plane-wave imaging (PWI).

The F-DMAS beamforming algorithm exploits the spatial coherence to enhance the image quality. In fact, there are many other ways to use the coherence besides the F-DMAS. One of them is to use the sign coherence factor (SCF) proposed by Camacho et al. [19] to weight the output of the DAS. It shows that this factor also can efficiently improve the resolution and contrast. The SCF is an extreme case of the phase coherence factor (PCF) [19]. The PCF can be considered as a weighting factor which is based on the phase consistency between signals. The backscattered signals from the focused point should have the same phase, and the consistency between out-of-focus signals is not good. Thus, we can use the statistical characteristics (standard deviation, variance, etc.) of the backscattered signals' phases to evaluate the quality of focusing. Based on the PCF, Hasegawa and Kanai [20] combined subaperture beamforming with phase coherence imaging, where the PCF is calculated in terms of the RF signals from the subapeture. In addition, there are several enhanced versions of PCF, such as exponential PCF, harmonic PCF, and Gaussian PCF [21].

In SCF, The received signals are divided into two polarities, positive and negative, according to different phases. SCF is calculated based on the statistical characteristic (standard deviation) of polarities. Then, the SCF is applied to weight the output of the DAS beamformer. However, because the polarity reflects the phase of the signal, one can also use a mean value of signals' polarities as a factor which we refer to as polarity-based factor (PF). Based on the F-DMAS and SCF, we proposed two new methods, the lag-based delay multiply and sum weighted by SCF (LAG-DMAS-SCF) and the lag-based delay multiply and sum weighted by PF (LAG-DMAS-PF). First, we construct a series of new signals based on the lag. The SCF and PF are then calculated from the new generated signals. Finally, the two factors are separately applied to weight the output of the DMAS beamformer.

The rest paper is organized as follows.  Section 2 mainly introduces the background. The detail of our proposed method is introduced in Section 3. The simulation and experimental results are exhibited in Section 4. After that, the discussion with respect to four beamformers is presented in Section 5. A brief conclusion is finally drawn in Section 6.

## 2. Background

### 2.1. Filtered-Delay Multiply and Sum (F-DMAS)

The algebra of DMAS algorithm is written as

(1) $$\begin{array}{c} y_{\text{DMAS}}=\overset{N-1}{\underset{i=1}{\sum }}\overset{N}{\underset{j=i+1}{\sum }}\mathrm{sign}\left(s_{i}s_{j}\right)∙\sqrt{\left|s_{i}s_{j}\right|}, \end{array}$$

where the *s*_*i*_ and *s*_*j*_ are the delayed signals received by the *i*^th^ and *j*^th^ element, respectively, and *N* is the total elements which are active in receiving. Due to the pair-wise multiplication, more frequency components exist in the final result. In order to retain the second harmonic component, the output of DMAS is passed through a bandpass filter to cancel the DC and higher frequency components. The sign, absolute, and square root operations in Equation (1) can be calculated previously using the following Equation (2) [15]:

(2) $$\begin{array}{c} {\bar{s}}_{i}=\mathrm{sign}\left(s_{i}\right)\sqrt{\;|\;s_{i}\;|\;},\text{for }1\leq i\leq N, \end{array}$$

Substituting Equation (2) into Equation (1), we can get

(3) $$\begin{array}{c} y_{\text{DMAS}}=\overset{N-1}{\underset{i=1}{\sum }}\overset{N}{\underset{j=i+1}{\sum }}{\bar{s}}_{i}{\bar{s}}_{j}. \end{array}$$

### 2.2. Sign Coherence Factor (SCF)

The SCF is an extreme form of PCF which utilizes the phases of received signals to evaluate the signal coherence [19]. In the SCF, the phase [−*π*, *π* ] is split into two intervals (−*π*/2,  *π*/2] and [−*π*, −*π*/2] ∪ (*π*/2, *π*]. The aperture data have thus only two polarities, positive or negative. Before evaluating the SCF, the polarity of each received signal needs to be decided by

(4) $$\begin{array}{c} b_{i}=\left\{\begin{array}{cc} -1, & s_{i}<0,\\ +1, & s_{i}\geq 0, \end{array}\right.\; \end{array}$$

where *s*_*i*_ is the delayed signal received by the *i*^th^ element. +1 means the positive polarity, and -1 means the negative polarity. The SCF can then be calculated by

(5) $$\begin{array}{c} \text{SCF}=1-\sqrt{1-{\left(\frac{1}{N}\overset{N}{\underset{i=1}{\sum }}b_{i}\right)}^{2}}, \end{array}$$

## 3. Method

The DMAS algebra can be expanded to

(6) $$\begin{array}{c} y_{\text{DMAS}}=\underset{\text{first item}}{\underset{⏟}{\left[{\bar{s}}_{1}{\bar{s}}_{2}+{\bar{s}}_{2}{\bar{s}}_{3}+\cdots +{\bar{s}}_{N-2}{\bar{s}}_{N-1}+{\bar{s}}_{N-1}{\bar{s}}_{N}\right]}}+\underset{\text{second item}}{\underset{⏟}{\left[{\bar{s}}_{1}{\bar{s}}_{3}+{\bar{s}}_{2}{\bar{s}}_{4}+\cdots +{\bar{s}}_{N-3}{\bar{s}}_{N-1}+{\bar{s}}_{N-2}{\bar{s}}_{N}\right]}}+\cdots +\;\underset{{\left(N-2\right)}^{\text{th}}\text{ item}}{\underset{⏟}{\left[{\bar{s}}_{1}{\bar{s}}_{N-1}+{\bar{s}}_{2}{\bar{s}}_{N}\right]}}+\underset{{\left(N-1\right)}^{\text{th}}\text{ item}}{\underset{⏟}{\left[{\bar{s}}_{1}{\bar{s}}_{N}\right]}}. \end{array}$$

Each item in Equation (6) is denoted by *x*_*l*_ for the sake of convenience:

(7) $$\begin{array}{c} x_{l}=\overset{N-l}{\underset{i=1}{\sum }}{\bar{s}}_{i}{\bar{s}}_{i+l},\text{for }1\leq l\leq N-1. \end{array}$$

The DMAS can then be re-written as

(8) $$\begin{array}{c} y_{\text{DMAS}}=\overset{N-1}{\underset{l=1}{\sum }}x_{l}. \end{array}$$

Here, *x*_*l*_ can be thought of as a new signal. Thus, the new signals (*x*_1_, *x*_2_ ⋯ *x*_*N*−1_) are sorted by the lag. Thanks to the relationship between the lag and spatial coherence [17], the new signals area also sorted by the spatial coherence. As with the expansion introduced in [22], the summation in Equation (8) is considered as a DAS operation. Therefore, a SCF can be used to weight its output. The corresponding polarity is then calculated by

(9) $$\begin{array}{c} b_{l}=\left\{\begin{array}{cc} -1, & x_{l}<0,\\ 1, & \;x_{l}\geq 0, \end{array}\right.\text{for }1\leq l\leq N-1. \end{array}$$

Let the SCF of the *x*_*l*_ be the SCF_LAG−DMAS_:

(10) $$\begin{array}{c} {\text{SCF}}_{\text{LAG}-\text{DMAS}}=1-\sqrt{1-{\left(\frac{1}{N-1}\overset{N-1}{\underset{l=1}{\sum }}b_{l}\right)}^{2}}. \end{array}$$

Multiplying the SCF_LAG−DMAS_ with *y*_DMAS_ get the final result *y*_LAG−DMAS−SCF_:

(11) $$\begin{array}{c} y_{\text{LAG}-\text{DMAS}-\text{SCF}}={\text{SCF}}_{\text{LAG}-\text{DMAS}}∙\overset{N-1}{\underset{l=1}{\sum }}x_{l}. \end{array}$$

Considering that the computational complex of SCF is somewhat high, we proposed another polarity-based factor (PF):

(12) $$\begin{array}{c} {\text{PF}}_{\text{LAG}-\text{DMAS}}=\frac{\;|\;\sum_{l=1}^{N-1}b_{l}\;|\;}{N-1}. \end{array}$$

This factor is actually an average value of all polarities. It can also reflect the phase diversity to a certain extent. Multiplying this factor with DMAS, we can get the final result *y*_LAG−DMAS−PF_:

(13) $$\begin{array}{c} y_{L\text{AG}-\text{DMAS}-\text{PF}}={\text{PF}}_{\text{LAG}-\text{DMAS}}∙\overset{N-1}{\underset{l=1}{\sum }}x_{l}, \end{array}$$

## 4. Results

The performance of four beamformers, DAS, F-DMAS, LAG-DMAS-PF, and LAG-DMAS-SCF, is compared. The software Field II [23, 24] is used to simulate several phantoms. Moreover, we also take into account the experimental and *in vivo* data.

In the simulation tests, a linear array with 128 elements and 38.4 mm width is modeled. In addition, the element width is 0.27 mm, element height is 5 mm, pitch size is 0.3 mm, and kerf is 0.03 mm. The elevation focus is at 30 mm. Two cycles of Hanning weighted sinusoidal excitation pulse is modeled, and the center frequency is 5 MHz. The sample frequency is 120 MHz. A low-pass filter is employed to remove the undesirable frequency components in the beamformed signals [25]. The numbers of elements, which are used to transmit and receive, are 32 and 64, respectively, and the transmission focal depth is 30 mm.

### 4.1. Simulated Point Targets

Twelve points are synthesized in the depth range from 15 mm to 40 mm with a 5 mm step, and there are 2 points at each depth. The lateral coordinates of two points at each depth are *x* = −1 mm and *x* = 1 mm, respectively.

The reconstructed images by DAS, F-DMAS, LAG-DMAS-PF, and LAG-DMAS-SCF are shown in Figure 1, respectively. The tailing at each point in Figure 1(a) is very severe. We cannot even distinguish between two points per depth. It means that the side lobe obtained by DAS should be very high. The smearing phenomenon can still be seen in Figure 1(b), but it is much better than Figure 1(a). Although the two points are not completely separated, we can, at least, see two points at each depth. In Figures 1(c) and 1(d), each point can be clearly observed, and two points at each depth are also completely separated. In addition, the smearing phenomenon cannot be observed in the two images. Compared to Figure 1(d), the points in Figure 1(c) are relatively larger. It means that the main lobe obtained by LAG-DMAS-PF is wider than LAG-DMAS-SCF.

Figure 2 depicts the lateral cross sections at three depths of 20 mm, 30 mm, and 40 mm, respectively. It can be seen from the figure that the main lobes and side lobes acquired by LAG-DMAS-PF and LAG-DMAS-SCF are respectively narrower and lower in comparison with DAS and F-DMAS. For example, at the depth of 40 mm, the side lobes obtained by DAS, F-DMAS, LAG-DMAS-PF, and LAG-DMAS-SCF are about -17 dB, -25 dB, -49 dB, and -69 dB, respectively. We can quantitatively compare the main lobe by FWHMs which are obtained by four algorithms at different depths. It can be seen from the Table 1, where the corresponding FWHMs are shown, that the values of LAG-DMAS-SCF are the best, followed by LAG-DMAS-PF, followed by F-DMAS, and the worst is DAS. This is also consistent with the results observed in Figures 1 and 2.

In the point target simulation, we can observe that applying a phase-related factor to weight the DMAS can get a better result. In the comparison between LAG-DMAS-PF and LAG-DMAS-SCF, the performance of LAG-DMAS-SCF is better.

### 4.2. Simulated Anechoic Cyst

A simulated anechoic cyst phantom is synthesized to evaluate the contrast of the images reconstructed by four algorithms. In a 20 × 20 × 1 mm^3^ volume, there are 200000 randomly distributed points which amplitudes follow the Gaussian distribution. An anechoic cyst with a radius of 4 mm is centered at (*x*,  *y*,  *z*) = (0,  0,  30) mm.

Figures 3(a)–3(d) show the reconstructed images by DAS, F-DMAS, LAG-DMAS-PF, and LAG-DMAS-SCF, respectively. The cysts in Figures 3(c) and 3(d) are much clearer than those in Figures 3(a) and 3(b). In Figure 3(a), the cyst is almost entirely blurred, with no edge visible. Compared to Figure 3(a), the situation in Figure 3(b) is slightly better; however, the cyst is still not clear. In Figure 3(c), the cyst is clear, and the edge can also be distinguished, but some smearing can be observed. Lastly, the cyst in Figure 3(d) is the clearest and the edge is also best defined. It is worth noting that there are some dark holes in the background in Figure 3(d). This may be a drawback of this method. Moreover, the lateral cross-section at the depth of 30 mm is shown in Figure 4 where we can see that the amplitude in the cyst obtained by LAG-DMAS-PF and LAG-DMAS-SCF is much lower than that of DAS and F-DMAS.

The contrast ratio (CR) which is normally used to quantitatively estimate the contrast is calculated by [6]:

(14) $$\begin{array}{c} \text{CR}=20\log_{10}\left(\frac{\mu_{\text{cyst}}}{\mu_{\text{bck}}}\right), \end{array}$$

where the *μ*_cyst_ and *μ*_bck_ are the mean intensities (before log-compression) of cyst (white box in Figure 3(a)) and background (black box in Figure 3(a)), respectively. The values of CR, obtained by DAS, F-DMAS, LAG-DMAS-PF, and LAG-DMAS-SCF, are -23.48 dB, -33.96 dB, -44.05 dB, and -60.51 dB, respectively. This also confirms the previous conclusion from the quantitative perspective.

### 4.3. Noise Influence Study

Noise is a very important factor affecting the quality of ultrasound images. Therefore, we try to evaluate the effects of the noise on the four algorithms. White Gaussian noise with SNR 10 dB is then added into the previous simulated point targets. The reconstructed images are shown in Figure 5.

In Figures 5(a) and 5(b), we can clearly see the effect of noise. In comparison, Figure 5(b) is slightly better than Figure 5(a) and shows a certain suppression of noise. However, in Figures 5(c) and 5(d), especially in Figure 5(d), the noise is effectively suppressed. Their corresponding lateral cross-sections at the depth of 20 mm, 30 mm, and 40 mm are shown in Figure 6. The FWHMs obtained by DAS, F-DMAS, LAG-DMAS-PF, and LAG-DMAS-SCF in a noisy environment at different depths are shown in Table 2 where the best values are highlighted in italics. There is no big difference from Table 1. In other words, the performance of LAG-DMAS-PF and LAG-DMAS-SCF is not affected even in an environment with relatively low SNR.

### 4.4. Experiment

In some cases, the contrast of target with respect to background may be not very high. The target is hard to detect accordingly. To evaluate the performance of four algorithms in these cases, we used a medical ultrasound machine iNSIGHT 37C (Saset, Chengdu, China) to get RF data by scanning a Multipurpose Multitissue ultrasound phantom (Model 040GSE. CIRS INC. 900 Asbury Ave Norfolk, Virginia 23513 USA). The center frequency and sampling frequency are 10 MHz and 60 MHz, respectively. The number of scan lines is 302. According to the phantom specification, the diameters of two gray scale targets, whose contrasts with respect to background are -9 dB and -6 dB, respectively, are both 8 mm.

The reconstructed images by the four beamformers are illustrated in Figure 7. The two targets are more detectable in Figures 7(c) and 7(d) than those in Figures 7(a) and 7(b). The two targets are blurred, and the edges are not distinguished in Figures 7(a) and 7(b). However, in Figure 7(d), the two targets, especially the right one, are clear and the edges are also well defined. Relatively speaking, the -6 dB target in Figure 7(c) is somewhat blurred, but the edges in Figures 7(c) can be clearly seen. The drawback in Figures 7(c) and 7(d) is that the dark holes can be observed, especially in Figure 7(d).

The corresponding values of CR evaluated using Equation (14) are depicted in Table 3. It shows that the LAG-DMAS-SCF gets the best contrast from quantity point of view. An interesting phenomenon is that the CRs obtained by F-DMAS and DAS are very close, and DAS is even better. This may be caused by some experimental parameters [26]. It means that the performance of F-DMAS may be vulnerable to these factors. But even in this case, LAG-DMAS-PF and LAG-DMAS-SCF still achieved significantly better results.

### 4.5. In Vivo

We also used the same ultrasound machine to scan the carotid artery. The number of scan lines is also 302. The reconstructed images are shown in Figure 8. In Figure 8(a), the carotid artery is hard to detect, and the lumen is totally blurred. It seems that the lumen in Figure 8(b) is more visible than that in Figure 8(a). Compared to Figures 8(a) and 8(b), the carotid arteries in Figures 8(c) and 8(d) are more detectable. The lumens in the two figures, especially in Figure 8(d), are clearer than those in Figures 8(a) and 8(b). In comparison with Figure 8(c), the carotid artery is more detectable in Figure 8(d). The shortage of Figure 8(d) is that the texture detail is weakened or even disappeared. Although this phenomenon can also be seen in Figure 8(c), it is not as severe as in Figure 8(d).

## 5. Discussion

In the DMAS beamforming algorithm, the signals are multiplied in pairs and then summed. If there are *N* signals, (*N*^2^ − *N*)/2 pair-wised signals are generated. These pair-wised signals can be rearranged in terms of lag. Summing the pair-wised signals with the same lag generates a new signal; then, we can get *N* − 1 new signals. Thereafter, the new synthesized signals are summed together to get the final result of DMAS. However, the process of summing new signals can be thought of as a DAS operation. As mentioned earlier, the DAS algorithm has certain limitations. Consequently, some coherence-based factors have been proposed to weight the output of DAS to get better image quality. It is very convenient to use a factor to weight the output of DAS, and calculating the factor is also simple. Considering that the final result of DMAS is the summation of new signals, we can also exploit a factor to weight its output. It should be noted here that the calculation of the factor in DMAS is based on new synthesized signals instead of those signals acquired by each element.

In our proposed methods, two factors, SCF and PF, are selected. As introduced earlier, the SCF and PF are both based on the polarity (or phase) of each signal; in our case, it is the polarity of each new synthesized signal. The spatial coherence is proportional to the autocorrelation of aperture function [27]. Compared to the signals from the elements that are far apart, signals from adjacent elements have higher coherence [17]. The spatial coherence has a close relationship with lag accordingly. From this point of view, the new generated signals are actually sorted by the coherence. Thus, the new signals can reflect the spatial coherence, and the coherence factor can be more appropriately evaluated.

The results show that the LAG-DMAS-PF and LAG-DMAS-SCF, in terms of resolution and contrast, outperform the DAS and F-DMAS. For a comparison between LAG-DMAS-PF and LAG-DMAS-SCF, the latter is better. However, compared to LAG-DMAS-PF, the dark hole phenomenon is more severe in LAG-DMAS-SCF. This may lead to the weakness of tissue structure. Therefore, if one wants to maintain the tissue structure as much as possible and hopes that the target can be better detected, the LAG-DMAS-PF is a good choice.

Compared to the original DMAS algorithm, there is only one more step to calculate the PF and SCF in LAG-DMAS-PF and LAG-DMAS-SCF, respectively. The computational complexity of SCF may be slightly high; however, the calculation of PF is really simple. Therefore, this point can also be used as a basis for choosing LAG-DMAS-PF or LAG-DMAS-SCF.

## 6. Conclusion

In this paper, we have presented two methods to improve the performance of the F-DMAS beamformer. The F-DMAS algorithm exploits the spatial coherence to enlarge the difference between the correlated signals and uncorrelated signals. Thus, we apply two phase coherence-related factors, which can also effectively reflect the spatial coherence, to enhance this feature. The results show that our proposed algorithms can improve the resolution and contrast to a certain extent.

## Figures and Tables

**Figure 1:** Images of simulated point targets reconstructed by (a) DAS, (b) F-DMAS, (c) LAG-DMAS-PF, and (d) LAG-DMAS-SCF. All images are shown in a dynamic range of 60 dB.

**Figure 2:** Lateral cross-sections in Figure 1 at the depth of (a) 20 mm, (b) 30 mm, and (c) 40 mm.

**Figure 3:** Images of simulated cyst reconstructed by (a) DAS, (b) F-DMAS, (c) LAG-DMAS-PF, and (d) LAG-DMAS-SCF. All images are shown in a dynamic range of 70 dB.

**Figure 4:** Lateral cross-section in Figure 3 at the depth of 30 mm.

**Figure 5:** Images of simulated point targets with white Gaussian noise (SNR = 10 dB) reconstructed by (a) DAS, (b) F-DMAS, (c) LAG-DMAS-PF, and (d) LAG-DMAS-SCF. All images are shown in a dynamic range of 60 dB.

**Figure 6:** Lateral cross-sections in Figure 5 at the depth of (a) 20 mm, (b) 30 mm, and (c) 40 mm.

**Figure 7:** Images of a tissue phantom reconstructed by (a) DAS, (b) F-DMAS, (c) LAG-DMAS-PF, and (d) LAG-DMAS-SCF. All images are shown in a dynamic range of 60 dB.

**Figure 8:** Images of a carotid artery reconstructed by (a) DAS, (b) F-DMAS, (c) LAG-DMAS-PF, and (d) LAG-DMAS-SCF. All images are shown in a dynamic range of 60 dB.

**Table 1:** FWHM (mm) at different depths in Figure 1.

Depth (mm)	Beamformer			
	DAS	F-DMAS	LAG-DMAS-PF	LAG-DMAS-SCF
15	0.48	0.32	0.22	*0.15*
20	0.55	0.36	0.31	*0.24*
25	0.50	0.35	0.31	*0.28*
30	0.67	0.41	0.36	*0.30*
35	0.80	0.53	0.38	*0.32*
40	0.91	0.67	0.49	*0.36*

**Table 2:** FWHM (mm) at different depths in Figure 5.

Depth(mm)	Beamformer			
	DAS	F-DMAS	LAG-DMAS-PF	LAG-DMAS-SCF
15	0.47	0.32	0.23	*0.17*
20	0.55	0.36	0.32	*0.28*
25	0.52	0.35	0.32	*0.28*
30	0.66	0.40	0.36	*0.30*
35	0.79	0.52	0.38	*0.29*
40	0.90	0.63	0.51	*0.34*

**Table 3:** CRs (dB) of two gray scale targets in Figure 7.

Gray scale target	Beamformer			
	DAS	F-DMAS	LAG-DMAS-PF	LAG-DMAS-SCF
Left	-8.72	-7.94	-13.75	*-18.53*
Right	-12.36	-11.30	-21.02	*-29.64*

## Data Availability

All data generated or analyzed during this study are included in this published article.
